The article "Research and Analysis of Brain Glioma Imaging Based on Deep Learning" was retracted in 2023. Reasons: signs of a paper mill; compromised peer review; unreliable results or conclusions.

# Research and Analysis of Brain Glioma Imaging Based on Deep Learning

**DOI:** 10.1155/2021/3426080

**Published:** 2021-11-18

**Authors:** Tao Luo, YaLing Li

**Affiliations:** ^1^Radiology Diagnostic Center, Hunan Cancer Hospital, Changsha 410000, China; ^2^Radiology Department, The Second People Hospital of Hunan Province, Changsha 410000, China

## Abstract

The incidence of glioma is increasing year by year, seriously endangering people's health. Magnetic resonance imaging (MRI) can effectively provide intracranial images of brain tumors and provide strong support for the diagnosis and treatment of the disease. Accurate segmentation of brain glioma has positive significance in medicine. However, due to the strong variability of the size, shape, and location of glioma and the large differences between different cases, the recognition and segmentation of glioma images are very difficult. Traditional methods are time-consuming, labor-intensive, and inefficient, and single-modal MRI images cannot provide comprehensive information about gliomas. Therefore, it is necessary to synthesize multimodal MRI images to identify and segment glioma MRI images. This work is based on multimodal MRI images and based on deep learning technology to achieve automatic and efficient segmentation of gliomas. The main tasks are as follows. A deep learning model based on dense blocks of holes, 3D U-Net, is proposed. It can automatically segment multimodal MRI glioma images. U-Net network is often used in image segmentation and has good performance. However, due to the strong specificity of glioma, the U-Net model cannot effectively obtain more details. Therefore, the 3D U-Net model proposed in this paper can integrate hollow convolution and densely connected blocks. In addition, this paper also combines classification loss and cross-entropy loss as the loss function of the network to improve the problem of category imbalance in glioma image segmentation tasks. The algorithm proposed in this paper has been used to perform a lot of experiments on the BraTS2018 dataset, and the results prove that this model has good segmentation performance.

## 1. Introduction

Brain tumor is an abnormal cell group that grows in brain tissue. This abnormal growth of cells seriously endangers human health. Compared with all cancer deaths, the mortality rate accounts for about 2.5% [1]. According to the location of origin, brain tumors are divided into two categories: the first category is primary brain tumors that originate in the brain, and the second category is secondary brain tumors that originate from malignant tumors outside the brain, but it has a spreading route. The starting point is to start from other parts of the body such as the digestive tract, liver, or breast and then invade into the skull. Among them, glioma is the most common primary brain tumor. It is caused by cancerous transformation of glial cell carcinoma of the brain and spinal cord, which accounts for more than 80% of malignant brain tumors [2]. In clinical practice, the location and type of glioma and the patient's physical health are the basis for judgment.

The article "Research and Analysis of Brain Glioma Imaging Based on Deep Learning" was retracted in 2023. Reasons: signs of a paper mill; compromised peer review; unreliable results or conclusions.

The size and shape of glioma are diverse, there are great differences among different patients, and it may occur anywhere in the brain. According to the patient's prognosis and the degree of invasion, gliomas are divided into high-grade gliomas and low-grade gliomas. Low-grade gliomas grow more slowly and patients have a longer survival period; relatively speaking, high-grade gliomas are more invasive and aggressive [3] and have a higher mortality rate and a shorter survival period. For glioma diseases, early and timely detection and detection of normal brain tissue lesions and targeted treatment improve the probability of patients being cured and are beneficial to human health. Therefore, how to effectively obtain the key information of glioma from medical images is the basis for reasonable treatment.

With the continuous development of modern medical imaging techniques, it provides important medical evidence for the diagnosis and treatment of glioma. Compared with computerized tomography (CT), magnetic resonance imaging (MRI) is often used clinically to detect and analyze brain gliomas. As we all know, in medical imaging methods, MRI has many advantages, such as high resolution and clear soft tissue structure. MRI is a noninvasive brain tumor imaging technology that is safe and harmless. It can provide clinicians with accurate information and become one of the important imaging technologies for the diagnosis and treatment of brain tumor diseases. From the imaging point of view, according to different imaging conditions, MRI brain images can be divided into four modes, namely, FLAIR mode, T1 mode, T1C mode, and T2 mode [4]. Since a single modality cannot fully express all the glioma areas, it may result in the loss of important glioma information. The glioma images based on multimodal MRI can better reflect gliomas' [5] specific location and shape; therefore, clinical radiologists usually combine four different modal images to comprehensively analyze and identify the area of glioma.

This paper studies how to use computer technology to automatically segment gliomas from normal brain tissues based on the image features in multimodal MRI images, so as to provide doctors with a basis for diagnosis and treatment. In this paper, MRI images of different modalities are used, fully combining the complementary advantages of different modal images to provide supplementary information for the analysis of different subregions of glioma, which can effectively improve the accuracy of segmentation.

The article "Research and Analysis of Brain Glioma Imaging Based on Deep Learning" was retracted in 2023. Reasons: signs of a paper mill; compromised peer review; unreliable results or conclusions.

## 2. Related Work

In recent years, segmentation algorithms based on deep learning have achieved good results and have attracted the attention of many scholars. Especially the combination of convolutional neural network (CNN) and computer vision field has made a key breakthrough in image segmentation [6].

Havaei et al. proposed a dual-path CNN model that uses different convolution kernels to extract global and local features, combined with multiscale features for brain tumor image segmentation, and the author also proposed a cascaded network, by combining an output of the branch network used as the input of another network to solve the problem of class imbalance [7]. Pereira et al. proposed a new network model based on the CNN model, using a small-sized convolution kernel to reduce network parameters, which can deepen the network level to obtain deeper feature information, obtained in the brain tumor segmentation challenge [8]. Ronneberger et al. proposed the earliest and most popular medical image semantic segmentation method “U-Net,” which is a fully convolutional network composed of two stages: contraction path and expansion path [9]. Iek et al. extended 2D U-Net to 3D U-Net and applied it to medical image segmentation to obtain richer spatial information of the image [10]. Liu Ping et al. proposed a deep-supervised DSSE-V-Net network model to automatically segment brain tumors. The network adds Squeeze-and-Excitation (SE) modules to the encoder and decoder paths to improve the V-Net model. The results show that the segmentation results of this model are stronger than the 3D U-Net and V-Net models [11]. Kamnitsas et al. achieved excellent results on BraTS2017 and proposed a segmentation method that integrates multiple models, called EMMA. This network combines DeepMedic [12] and U-Net model to integrate their details, subprediction [13]. In 2018, Myronenko et al. proposed a 3D codec model based on ResNet and won the first prize in BraTS2018 [14]. Zhou et al. integrated several different networks and used shared weights to extract multiscale context information [15]. Chu et al. designed a two-classification network based on cascade, which separately segmented the three brain tumor subregions, and merged the results to generate the final result [16]. Huo et al. designed a dual-channel dense connection network based on the differences in the location and shape of brain tumors, thereby extracting image features through multiscale convolution kernels [17]. Khan et al. proposed an automatic multimodal classification method that uses deep learning to classify brain tumor types [18]. The method includes five core steps. The first step uses edge-based histogram equalization and discrete cosine transform (DCT) for linear contrast stretching; the second step uses transfer learning to use two pretrained CNN models VGG16 and VGG19 for feature extraction. The third step is to use a correlation-based joint learning method combined with an extreme learning machine (ELM) for feature selection. The fourth step is to fuse robust covariant features based on partial least squares (PLS) into a matrix. The combined matrix is sent to ELM for the final multimodal brain tumor classification. Zhou et al. designed a three-stage network: generation constraints, constrained fusion, and final segmentation. First, in the 3D U-Net segmentation network, additional context constraints are generated for each tumor region; second, under the obtained constraints, the attention mechanism is used to fuse multisequence MRI to achieve the segmentation of three subtumor regions; finally, 3D U-Net model combines and refines the above prediction results [19]. Rehman et al. proposed a two-dimensional image segmentation method (BU-Net), which incorporates a residual extended skip (RES) module and a wide context (WC) module based on the U-Net network. Aggregated features are used to extract contextual information to obtain better segmentation performance [20]. Luo et al. designed a lightweight but efficient HDC-Net model to solve the segmentation problem of brain tumors. In order to reduce computational overhead, the author designed a new type of hierarchical decoupled convolution (HDC) module, which can efficiently explore multiscale, multiview spatial context and reduce the number of parameters [21]. Li et al. proposed a brain tumor segmentation method based on Generative Adversarial Networks (GAN). The network architecture consists of a densely connected 3D U-Net model for segmentation and a classification network for discrimination. Both use three-dimensional convolution to fuse multidimensional context information [22]. Although the deep learning-based automatic segmentation algorithm for glioma has achieved good results, there are still challenges to accurately achieve the automatic segmentation task of glioma. The main reasons are as follows. (1) Glioma has antenna-like structure often spreading easily and having poor contrast. (2) There are diversified positions, shapes, and sizes of gliomas, and there are very big differences among different patients. (3) Gliomas blurred boundaries with surrounding tissues. The existence of these factors makes it extremely difficult to accurately segment gliomas.

The article "Research and Analysis of Brain Glioma Imaging Based on Deep Learning" was retracted in 2023. Reasons: signs of a paper mill; compromised peer review; unreliable results or conclusions.

## 3. Method

### 3.1. Algorithm Overview

The MRI-based automatic segmentation algorithm for glioma needs to determine the location of each area of the glioma. Therefore, a method based on fully convolutional neural network is proposed to realize the segmentation of glioma. In view of the fact that 3D U-Net is widely used in medical image segmentation to obtain good segmentation results, this section uses the 3D U-Net model for glioma image segmentation, which has problems such as insufficient detail segmentation and unclear boundary segmentation. The problem improved this network. In this section, a new brain glioma segmentation network is designed, called Dilated Dense Block-UNet (DDB-UNet) based on the hollow dense block.

The DDB-UNet model mainly consists of three different structures. The first part is the encoder-decoder structure. The second part is the Dense Dilated Block (DDB) proposed by the network. Finally, a mixed loss function is used to constrain the proposed network, which can speed up the convergence speed of the network model. DDB-UNet makes full use of the jump connections and densely connected blocks of the 3D U-Net model [23] to improve the ability to acquire image features, extract rich context information, and expand the receptive field of the convolution kernel by using hole convolution [24].

### 3.2. Algorithm Framework Description

#### 3.2.1. Basic Network

The 3D U-Net model is expanded based on the 2D U-Net model and is used in the segmentation of 3D images. In this section, the input channel is set to 4, corresponding to four modal MRI images. The 3D U-Net model consists of two parts, the encoding part and the decoding part.

Among them, the coding part is composed of three submodules. Each submodule includes two 3 × 3 × 3 convolutional layers. After two convolution operations, they are operated by Batch Normalization and ReLU activation function and used by 3D U-Net. Batch Normalization is used to make the network better converge and speed up the training speed of the model. Through experiments, it is found that Batch Normalization can also improve the segmentation effect of the model. As an activation function, ReLU is used to add nonlinear factors between the layers of the neural network to overcome the problem of vanishing gradients. The coding part also includes three downsampling, and each downsampling module uses a 2 × 2 × 2 maximum pooling layer with a step size of 2. With the continuous deepening of the network model, the number of model parameters has increased rapidly. Using the Batch Normalization layer on the network can solve the phenomenon of gradient disappearance. The function of the coding part is to analyze the entire image and extract spatial information. The decoding part includes three submodules, each of which includes upsampling. The upsampling module consists of a 2 × 2 × 2 deconvolution layer with a step length of 2, followed by two 3 × 3 × 3 convolutional layers, through the Batch Normalization and ReLU activation functions. The function of the decoding part is to restore the downsampling and reduced feature map to the same size as the input image through the upsampling operation, and the resolution is sequentially increased through the upsampling operation until it is consistent with the resolution of the input image, and the target area is located. The last layer is a 1 × 1 × 1 convolution, which can reduce the number of output channels, and the final output channel number is the number of label categories. 3D U-Net uses skip connections to connect the upsampling feature map of the decoding part with the output of the submodule with the same resolution in the encoding part, as the input of the next submodule in the decoding part, combining low-level features and high-level features fusion, so as to achieve the purpose of optimizing the output results.

The article "Research and Analysis of Brain Glioma Imaging Based on Deep Learning" was retracted in 2023. Reasons: signs of a paper mill; compromised peer review; unreliable results or conclusions.

#### 3.2.2. Hole Convolution

In recent years, it has been shown from deep learning research that the increase in the receptive field of the convolution filter is very meaningful for extracting more spatial information [25]. The pooling layer is usually used to expand the receptive field, but the pooling layer operation will reduce the size of the feature map and restore the size of the image through upsampling. This may lead to the loss of some spatial information. In order to solve the above problems, Yu et al. proposed a hole convolution, whose purpose is to increase the receptive field while keeping the size of the feature map unchanged.

The hole convolution replaces the original convolution, and holes are injected into the standard convolution kernel to increase the receptive field. To improve the accuracy of segmentation in the segmentation task of glioma based on the fully convolutional neural network, this section uses the hollow convolution to expand the feature receptive field of the network model and obtain more detailed information of the glioma. The difference between the hole convolution and the ordinary convolution is that the hole convolution has a parameter called the expansion rate, which represents the distance between adjacent elements in the hole convolution kernel. The cavity convolution obtains information of different scales according to different expansion rates, expands the receptive field of the filter without increasing the amount of parameters and calculations, and obtains more characteristic information of glioma. The advantage of hollow convolution is that without adding additional calculation parameters, different expansion rates are set in each convolution to obtain different sizes of receptive fields, which can complete the exchange of global information between layers. The network structure based on hole convolution can obtain multiscale context information.

The article "Research and Analysis of Brain Glioma Imaging Based on Deep Learning" was retracted in 2023. Reasons: signs of a paper mill; compromised peer review; unreliable results or conclusions.

#### 3.2.3. Densely Connected Block

At present, in order to obtain more advanced and abstract feature information, the designed deep learning network model is continuously deepened to improve the accuracy. In the actual training process, as the network depth continues to increase, the network is more difficult to train, resulting in a decrease in the generalization ability of the model. Positively influenced by the idea of residual network, Huang et al. proposed the DenseNet network model, which became the best paper of the year [23]. The learning strategy is similar to the residual network, and the module structure has been modified, which greatly increases the width of the identity mapping. The overall structure is similar to the U-Net network model structure. Both are based on the segmentation model of the fully convolutional neural network, including the downsampling module and the upsampling module, and the whole is U-shaped. The difference is that the densely connected block in DenseNet has higher feature map reuse characteristics. The input data of each convolution block in the densely connected block contains the output data of all previous convolutional blocks, which can be effective. Use the information of the feature map to enhance the transmission of information, so that the features extracted by the network can contain both low-level location information and high-level semantic information. The dense connection block incorporated in this section is to expand the dense connection block in DenseNet into a three-dimensional structure, which is helpful to obtain the spatial information of the MRI glioma image.

Figure 1 shows the structure of densely connected blocks. In order to improve the information transfer of feature maps between layers, in the dense connection block, different connection modes are designed, from any layer to all subsequent layers directly connected. These additional connections are called dense connections, which help gradients flow and allow the network to extract richer features. In the densely connected block, the input of each convolutional layer will be merged with all the previous layers in the feature dimension and used as the input of the next layer.

The article "Research and Analysis of Brain Glioma Imaging Based on Deep Learning" was retracted in 2023. Reasons: signs of a paper mill; compromised peer review; unreliable results or conclusions.

The output of each convolution block in the densely connected block is used as the input of the next convolution block, which strengthens the information transfer between the convolution blocks. Densely connected blocks are used to extract local context information, which makes the network extract richer multilevel features. The dense connection block used in this section is a basic module in DenseNet. Densely connected blocks have a larger model capacity than conventional convolutional blocks. DenseNet is suitable for training larger data and has a strong generalization ability.

#### 3.2.4. Hollow Dense Module

In order to enhance the information transfer of feature maps between layers, densely connected blocks are introduced into the model. At the same time, in order to expand the receptive field, an expansion rate is added to each densely connected block. The size of each convolution kernel is finally designed to be 3 × 3 × 3. The densely connected block is integrated into U-Net to enhance the connection between layers, and the expansion of densely connected blocks to three-dimensional structures helps to better extract the spatial information of three-dimensional MRI gliomas. In the densely connected block, the three parts of Batch Normalization, ReLU nonlinear activation function, and 3 × 3 × 3 convolution block form a layer of convolution block structure, and the input of each convolution block contains all the previous convolutions. The output of the product block can reuse the feature map, strengthen the information flow between convolution blocks, reduce the amount of parameters, alleviate the problem of gradient disappearance, and make the forward propagation of features and the backward propagation of gradients more effective.

The hollow dense module not only expands the receptive field but also promotes the transfer of information between layers. We innovatively use dense connection blocks to efficiently reuse feature maps and improve the feature extraction capabilities of the network. To expand the receptive field while keeping the input feature dimension unchanged, we add an expansion rate to each densely connected block. Therefore, the receptive field is expanded by hollow convolution to capture contextual information, and densely connected blocks maximize the information flow between layers and improve the feature extraction ability of the network.

### 3.3. 3D U-Net Structure Based on Hollow Dense Blocks

The 3D U-Net algorithm has achieved good segmentation results in the field of medical image segmentation, but there are some problems in applying the 3D U-Net structure to the segmentation task of glioma, such as insufficient segmentation of the glioma boundary. The details of the glioma are not well represented. In this section, in view of the insufficient detail segmentation of the 3D U-Net algorithm in the segmentation of glioma images, the 3D U-Net algorithm is improved on the basis of further improving the results of glioma segmentation, and a method based on holes is proposed, Dense block 3D U-Net structure (DDB-UNet). The model takes four modal MRI glioma images as input, and the network structure is shown in Figure 2.

The article "Research and Analysis of Brain Glioma Imaging Based on Deep Learning" was retracted in 2023. Reasons: signs of a paper mill; compromised peer review; unreliable results or conclusions.

In the segmentation of brain glioma, in view of the uncertainty of the location and area of brain glioma, the diversity of size and shape makes the task of segmentation of brain glioma challenging. This section proposes to add hollow convolution to the network structure to improve the receptive field of the original model so that through the characteristics of glioma we can obtain more abstract feature information in the deep layer of the network. In this section, inspired by the DenseNet network structure, densely connected blocks are applied to the 3D U-Net model to achieve efficient use of feature maps, so that the network can obtain rich multiscale feature information and better solve the brain glial problem of unclear segmentation of tumor image boundary. Densely connected blocks are used instead of ordinary convolution blocks, which can enhance the information exchange between the layers of the feature map and improve the feature extraction ability of the network. The expansion rate is added to the dense connection block to construct a hollow dense module, which not only expands the receptive field but also promotes the transfer of information between layers. The 3D DDB-UNet segmentation network designed in this section is composed of two parts: (1) the overall framework, a 3D U-Net model, and (2) Hole Dense Module (DDB). The purpose of the 3D DDB-UNet model is to effectively combine the respective advantages of the cavity module and the densely connected module, so that the performance of the network model in the segmentation process of glioma can be further improved.

### 3.4. Loss Function

The loss function is to measure the gap between the true label value and the predicted value. Constraining the network during the training process and optimizing network parameters can enable the network to obtain more meaningful features. According to the segmentation work of glioma, in the entire MRI image, the target glioma area accounts for a very small proportion, and there is a serious imbalance between the glioma area and the background area. Milletari et al. proposed the Dice loss function in 2016 and applied it to the image segmentation task. Using the Dice loss function in the binary classification problem can effectively alleviate the problem of category imbalance, but there will be some defects in the multiregion segmentation work [26]. In the training task, it will cause the training to be unstable. Sudre et al. proposed the Generalized Dice Loss (GDL) loss function for multiclassification tasks [27]. GDL integrates the Dice results of multiple categories and quantifies the results obtained by segmentation. The expression is as follows:

(1) $$\begin{array}{c} L_{\text{GDL}}=1-\frac{2\sum_{i=1}^{m}w_{i}\sum_{j=1}^{N}r_{ij}p_{ij}}{m\sum_{i=1}^{m}w_{i}\sum_{j=1}^{N}\left(r_{ij}+p_{ij}\right)}. \end{array}$$

In the model of this paper, GDL is used as the loss function. In addition, on the basis of the GDL loss function, the cross-entropy loss function is added in order to strengthen the model's learning of multiple targets in the region as follows:

(2) $$\begin{array}{c} L_{CE}=-\sum_{j=1}^{v}r_{j}\log\;p_{j}. \end{array}$$

The loss function used in this section consists of two parts: one is the multiclass Dice loss function GDL, and the other is the cross-entropy loss function between the predicted result and the real label. The final loss is expressed as

(3) $$\begin{array}{c} \text{Loss}=L_{\text{GDL}}+L_{\text{CE}}. \end{array}$$

The article "Research and Analysis of Brain Glioma Imaging Based on Deep Learning" was retracted in 2023. Reasons: signs of a paper mill; compromised peer review; unreliable results or conclusions.

## 4. Experiments and Discussions

### 4.1. Dataset

The data used in this paper comes from the multimodal brain tumor segmentation challenge BraTS2018. There are two types of data in the BraTS2018 dataset: high-grade glioma and low-grade glioma. There are 210 samples of high-grade glioma and 75 samples of low-grade glioma. Each case sample is three-dimensional data, and each case contains four modal MRI glioma images and ground truth label maps, of which the four modalities are FLAIR, T1, T1C, and T2. The truth-value label map was manually annotated by a number of experts according to the outline of the tumor. The size of each mode is 155 × 240 × 240; that is, there are 155 pictures with a size of 240 × 240, and the total data volume of each sample is 4 × 155 × 240 × 240. The data of each case is divided into five categories at the voxel level: necrosis, edema, enhancement, nonenhanced tumor, and normal tissue.

### 4.2. Evaluation Metric

In the segmentation task of brain glioma, the three indicators of Dice, PPV, and sensitivity are often used to evaluate the performance of brain glioma segmentation. The calculation is as follows:

(4) $$\begin{array}{c} \text{Dice}=\frac{2TP}{FP+2TP+FN},\\ \text{PPV}=\frac{TP}{TP+FP},\\ \text{sensitivity}=\frac{TP}{TP+FN}. \end{array}$$

The article "Research and Analysis of Brain Glioma Imaging Based on Deep Learning" was retracted in 2023. Reasons: signs of a paper mill; compromised peer review; unreliable results or conclusions.

### 4.3. Optimization Verification of Loss Function

This section uses experiments to verify whether the multiclass loss function (GDL) and cross-entropy loss function (CE) in the proposed algorithm can improve the performance of glioma segmentation. The experiments are as follows: experiment one: DDB-UNet model + GDL loss function; experiment two: DDB-UNet model + CE loss function; and experiment three: DDB-UNet model + GDL loss function + CE loss function. The experimental results are shown in Table 1 and Figures 3–5, where WT represents the complete tumor area, TC represents the core tumor area, and ET represents the enhanced tumor area.

As illustrated in Table 1, by showing the segmentation results of different loss functions in the BraTS2018 dataset, the following conclusions can be drawn. (1) The experimental results obtained by using the GDL loss function and the Cross-Entropy loss function in the DDB-UNet model are the best of all the above methods and the evaluation index of this method is the highest. (2) Integrating the two loss functions of GDL loss function and Cross-Entropy loss function into the network model can alleviate the class imbalance problem in the segmentation of glioma images and use these two loss functions to separate the network model. The impact is not big, but combining these two loss functions, the segmentation performance of the network model is relatively obvious. Therefore, the experimental results can show that the use of a hybrid loss function combining the GDL loss function and the Cross-Entropy loss function restricts the network model training and improves the segmentation performance of the network model. (3) The GDL loss function and the Cross-Entropy loss function alleviate the class imbalance problem in glioma image segmentation to a certain extent and get a good network segmentation effect. Therefore, this paper uses the hybrid loss function combined with the GDL loss function and the Cross-Entropy loss function to train the network model.

### 4.4. Comparison of Algorithm Performance

In Table 2, the Dice values of different segmentation algorithms are compared. By comparing the Dice results of different segmentation networks in Table 2, compared with the basic network 3D U-Net, the network designed in this section has a Dice value in the segmentation tasks of the complete tumor region, core tumor region, and enhanced tumor region getting significant improvement. Compared with other algorithms, in the task of segmenting smaller regions, the result of designing the network in this section is the best.

The experimental results can show that the segmentation results of the DDB-UNet network model proposed in this section are the best among the above network models. The Dice values of the complete tumor area, core tumor area, and enhanced tumor area have reached the best performance. Whether it is the most advanced segmentation method, or compared with the 3D U-Net method, there is a significant improvement.

The article "Research and Analysis of Brain Glioma Imaging Based on Deep Learning" was retracted in 2023. Reasons: signs of a paper mill; compromised peer review; unreliable results or conclusions.

## 5. Conclusions

The object of this study is glioma, which is one of the most common brain tumors with a very high fatality rate. In the clinic, doctors manually segment glioma images based on clinical experience, which not only consumes a lot of time and energy, but also is easily affected by the doctor's subjectivity. Therefore, the study of an automatic segmentation technology for MRI glioma images can help doctors formulate a diagnosis plan and has very important research value for the diagnosis and treatment of glioma. This paper is based on deep learning algorithms to process MRI glioma images and complete the automatic segmentation of glioma images. The main research contents are as follows: propose a glioma segmentation model (DDNet) based on 3D U-Net with dense blocks of holes. On the basis of the U-Net network structure, the hollow convolution and dense convolution are integrated into it. Each layer of the U-Net network is composed of the hollow convolution and densely connected blocks. When training the network model, the multiclass loss function and the cross-entropy loss function are used to optimize the performance of the network and alleviate the class imbalance problem in the segmentation of glioma. Finally, a variety of evaluation indicators are used to verify the effectiveness of the network model based on dense blocks of holes proposed in this section for segmentation of glioma images.

## Figures and Tables

**Figure 1:** Schematic diagram of densely connected blocks.

**Figure 2:** DDB-UNet segmentation model.

**Figure 3:** Segmentation results for Dice.

**Figure 4:** Segmentation results for sensitivity.

**Figure 5:** Segmentation results for PPV.

**Table 1:** Segmentation results of different loss functions.

Loss	Dice			Sensitivity			PPV		
	WT	TC	ET	WT	TC	ET	WT	TC	ET
GDL	0.864	0.817	0.772	0.885	0.818	0.781	0.883	0.887	0.753
CE	0.872	0.820	0.777	0.891	0.826	0.792	0.887	0.893	0.768
GDL + CE	0.886	0.824	0.787	0.893	0.894	0.801	0.898	0.900	0.779

**Table 2:** Comparison of dice effects of different algorithms.

Method	Dice		
	WT	TC	ET
3D U-Net	0.885	0.769	0.719
Dense-UNet	0.876	0.821	0.771
VAE-Encoder	0.883	0.814	0.767
S3D-UNet	0.881	0.809	0.734
OM-Net	0.877	0.756	0.660
Ours	0.886	0.824	0.787

## Data Availability

The datasets used and analyzed during the current study are available from the corresponding author upon reasonable request.
